The article "The influence of vermicomposting on photosynthetic activity and productivity of maize (Zea mays L.) crop under semi-arid climate" was retracted in 2022. Reasons: compromised peer review; a conflict of interest; concerns about the authorship.

# The influence of vermicomposting on photosynthetic activity and productivity of maize (*Zea mays* L.) crop under semi-arid climate

**DOI:** 10.1371/journal.pone.0256450

**Published:** 2021-08-25

**Authors:** Muhammad Younas, Huasong Zou, Tasmia Laraib, Waseem Abbas, Muhammad Waqar Akhtar, Muhammad Naveed Aslam, Luqman Amrao, Shoukat Hayat, Tariq Abdul Hamid, Akhtar Hameed, Ghalib Ayaz Kachelo, Mona M. Elseehy, Ahmed M. El-Shehawi, Ali Tan Kee Zuan, Yunzhou Li, Muhammad Arif

**Affiliations:** 1 Department of Plant Pathology, College of Agriculture, Guizhou University, Guiyang, Guizhou, China; 2 Department of Plant Pathology, University of Agriculture Faisalabad, Punjab, Pakistan; 3 College of Plant Protection, Fujian Agriculture and Forestry University, Fujian, Fuzhou, China; 4 Institute of Molecular Biology and Biotechnology, The University of Lahore, Lahore, Punjab, Pakistan; 5 Ayub Agricultural Research Institute, Faisalabad, Punjab, Pakistan; 6 Department of Soil Science, The Islamia University of Bahawalpur, Bahawalpur, Punjab, Pakistan; 7 Department of Plant Pathology, The Islamia University of Bahawalpur, Bahawalpur, Punjab, Pakistan; 8 Department of Forestry, Department of Forestry, The Islamia University of Bahawalpur, Bahawalpur, Punjab, Pakistan; 9 Assistant Director, office of Deputy Director of Agriculture, Pest Warning & Quality Control of Pesticides (PW&QCP) Lahore, Lahore, Pakistan; 10 Department of Genetics, Faculty of Agriculture, University of Alexandria, Alexandria, Egypt; 11 Department of Biotechnology, College of Science, Taif University, Taif, Saudi Arabia; 12 Department of Land Management, Faculty of Agriculture, Universiti Putra Malaysia, Serdang, Selangor, Malaysia; 13 Department of Plant Protection, Fujian Agriculture and Forestry University, Fuzhou, China; Ghazi University Dera Ghazi Khan, PAKISTAN

## Abstract

Food production and waste recycling are the two major issues faced globally with rapidly increasing population. Recycling organic wastes to crop amendments could be a possible solution to these issues. Earthworms transfer organic waste to compost, which is used to grow crops and increase crop productivity. This study assessed the impact of vermicompost produced from the residues of six desert plant species, i.e., (*Ziziphus mauritiana*, *Aerva javanica*, *Calligonum comosum*, *Sacchrum benghalens*, *Calligonum polygonoides* and *Prosopis cineraria*) combined with farmyard manure (5 t ha^-1^) on growth, yield and photosynthetic activity of maize crop. Earthworm species *Eisenia fetida* (Savigny, 1826) was used to prepare vermicomposting of all tested plant species. The desert species were collected from natural habitats, chopped, dried, mixed with FYM and then earthworms were released to prepare the vermicompost. The earthworms were excluded twenty days after release and resultant was considered as compost and used in the experiment. Results revealed that application of *P*. *cineraria* vermicompost resulted in the highest plant height (75.33 cm), stem diameter (22.66 mm), cob length (17.66 cm), number of grains/cob (374.67), 1000-grain weight (260.41 g) and grains yield (3.20 t/ha). Application of *P*. *cineraria* vermicompost resulted in the highest uptake of macronutrients, i.e., N (91.01%), P (22.07%), K (80.41%), micronutrients, i.e., Fe (19.07 ppm), Zn (40.05 ppm), and phenolic contents (150). Application of *P*. *cineraria* vermicompost also resulted in the highest quantum photosynthetic yield (0.42 mole C/mole of photon), chlorophyll florescence (355.18 moles of photon m^-2^s^-1^) and electron transport rate (310.18 micro mole m^-2^s^-1^). It is concluded that vermicomposting has the potential to improve growth and yield of maize crop. Particularly, application of vermicompost obtained from *P*. *cineraria* can be used to improve the growth and yield of maize crop. Nonetheless, field trials are necessary for a wide scale recommendation.

The article "The influence of vermicomposting on photosynthetic activity and productivity of maize (Zea mays L.) crop under semi-arid climate" was retracted in 2022. Reasons: compromised peer review; a conflict of interest; concerns about the authorship.

## Introduction

Conventional agriculture is reliant on excessive application of pesticides, herbicides, chemical fertilizers and low use of organic fertilizers [1, 2]. Frequent and non-judicious application of chemicals exerts various negative effects on environment [3], causes food pollution [4, 5], decreases soil quality and results in the loss of agricultural biodiversity [6–8]. Sustainable agricultural practices relying on natural or organic sources are needed to overcome these hazards.

Organic farming is the widely accepted option for maintaining the environmental sustainability and biodiversity [9, 10]. Organic farming is being adopted by the environment-sensitive populations in developed countries due to its enormous ecological and economic benefits [11, 12]. Previous studies revealed that vermicomposting improves nutrient status as well as biological characters of soil [13]. It is highly beneficial as it allows good drainage, improves water storage capacity and soil ventilation [14].

The production of livestock manure has been considerably increased due to rapidly increasing industrialization and human population [15, 16]. However, it caused numerous environmental drawbacks including contaminated ground water and offensive odors [17, 18]. The conversion of waste to valuable materials may could play a significant role in environmental cleaning and resource recycling [19]. Various microbiological, physical and chemical techniques are used for the disposal of livestock manure. Unfortunately, all these strategies are labor intensive and time-consuming [20–23]. Traditional composting is cheap and unadorned; however, it causes nutrient losses [24, 25].

The article "The influence of vermicomposting on photosynthetic activity and productivity of maize (Zea mays L.) crop under semi-arid climate" was retracted in 2022. Reasons: compromised peer review; a conflict of interest; concerns about the authorship.

Vermicomposting is a viable and cost effective technique for the management of livestock manure. Earthworms’ activity initiates the decomposition of organic matter and prepares nutrients for plant growth [26, 27]. Thus, composting of livestock manure is helpful in reducing environmental pollution and also provides a healthier substitute of chemical fertilizers [28]. Studies relating to photosynthesis in maize crop are important for the selection of superior genotypes and improve yield under abiotic stresses [29, 30]. Chlorophyll fluorescence and electron transport rate directly influence plant vegetative growth, which ultimately leads to higher yield [31].

Although several studies have reported the benefits of vermicomposting, rare studies have combined plant residues and FYM to produce a nutrient rich compost. Therefore, this study produced compost of FYM combined with plant residues and tested their impacts on growth, photosynthesis and yield of maize crop. The major aim of the study was to select the most suitable desert species for vermicomposting. Investigate the impacts of applied vermicompost on the yield of maize crop was the second objective of the study.

## Materials and methods

### Experimental site

The experimental site is located at Students Research Farm, University of Agriculture Faisalabad, Pakistan (31.4278° N, 73.0758° E). The climate of the study area is semi-arid. The average temperature is 24.8°C, while annual rainfall is 526 mm. Soil type is silt-loam to sandy-loam. Physio-chemical properties of soil were determined before the initiation of experiment and are given in Table 1.

**Table 1:** Physio-chemical parameters of experimental soil.

Soil properties	Values
Total nitrogen (%)	0.038
Organic matter (%)	0.77
pH	8.4
Electric conductivity (mS cm^-1^)	1.35
Available potassium (%)	160
Available phosphorus (%)	7.2
Textural class	Loam

### Experimental design

Six desert plant species, i.e., *Ziziphus mauritiana*, *Aerva javanica*, *Calligonum comosum*, *Sacchrum benghalens*, *Calligonum polygonoides* and *Prosopis cineraria* were collected from the surroundings of Faisalabad and Bhakkar, Pakistan. Similarly, farmyard manure (FYM) was collected from Student Research Farm, University of Agriculture, Faisalabad, Pakistan. Collected materials were dried and crushed at biogas plant located at Research farm, University of Agriculture, Faisalabad, Pakistan. After processing, the material was mixed with FYM and soil. Twenty individuals of earthworm [*Eisenia fetida* (Savigny, 1826)] were added into each pot and kept wet for twenty days [32]. The earthworms were discarded by following the sieve method and vermicompost was transferred to pots (Table 2). Maize plants were grown in the pots. Experiment was laid out by following the complete randomized design. The treatments used in the experiment are given in Table 2.

The article "The influence of vermicomposting on photosynthetic activity and productivity of maize (Zea mays L.) crop under semi-arid climate" was retracted in 2022. Reasons: compromised peer review; a conflict of interest; concerns about the authorship.

**Table 2:** Experimental treatments used in the study, their abbreviations and explanations.

Abbreviation	Treatments
T_0_	Absolute control*
T_1_	Vermicompost of *Ziziphus mauritiana* + FYM* *
T_2_	Vermicompost of *Aerva javanica* + FYM
T_3_	Vermicompost of *Calligonum comosum* + FYM
T_4_	Vermicompost of *Sacchrum benghalens* + FYM
T_5_	Vermicompost of *Calligonum polygonoides* + FYM
T_6_	Vermicompost of *Prosopis cineraria* + FYM

*The plants were grown on simple soil,

**Five tons per hectare farmyard manure (FYM) was added

### Photosynthetic yield analyzer

Photosynthetic yield analyzer was used to measure the photosynthetic efficiency of photosystem II and physiological parameters of photosystem II, including, quantum photosynthetic yield (mol C/mole of photon), chlorophyll florescence (moles of photons m^-2^/S) and electron transport rate (μmolm^-2^S^-1^). The Kjeldahl and Champ and Marker method [33] was used for determining the nitrogen, phosphorus and potassium. This Kjeldahl method is mainly divided in three steps, i.e., digestion, distillation and titration. Homogenous samples were boiled in concentrated sulfuric acid, which lead to the formation of ammonium sulfate solution. Excess base was added for converting NH_4_ to NH_3_ and then amount of nitrogen was calculated from the ammonia [34].

### Determination of micronutrients

Atomic absorption spectrophotometer (Hitachi Polarized Zeeman AAS, Z-8200, Japan) was used for determining the minerals, i.e., iron (Fe) and zinc (Zn) following the conditions described in AOAC. The instrumental operating conditions are summarized in Table 3.

**Table 3:** Operational conditions used in atomic absorption spectrophotometer for the determination of iron (Fe) and zinc (Zn).

Parameters	Set value	
	Fe	Zn
Wavelength (nm)	248.3	213.9
Slit Width (nm)	0.2	1.3
Lamp Current (mA)	10.0	10.0
Burner Head	Standard type	Standard type
Flame	Air-C_2_H_2_	Air-C_2_H_2_
Burner Height (mm)	7.5	7.5
Oxidant gas pressure (Flow rate) (kpa)	160	160
Fuel gas pressure (Flow rate) (kpa)	6	6

### Standards’ preparation

Calibrated standards were prepared from the commercially available stock solution (AppliChem^®^) in the form of aqueous solution (1000 ppm). Highly purified de-ionized water was used for the preparation of working standards. All the glass apparatus used throughout the process of analytical work were immersed in 8N HNO_3_ overnight and washed with several changes of de-ionized water prior to use.

The article "The influence of vermicomposting on photosynthetic activity and productivity of maize (Zea mays L.) crop under semi-arid climate" was retracted in 2022. Reasons: compromised peer review; a conflict of interest; concerns about the authorship.

### Statistical analysis

The data were recorded using the standard procedures and statistically analyzed at 5% level of significance using Fisher’s analysis of variance (ANOVA) technique. One-way ANOVA was used to test the significance among treatments and data were normalized prior to execute ANOVA. The treatment means were compared using least significant different test as a post-hoc test where ANOVA indicated significant differences [35].

## Results and discussion

### Growth and yield attributes

Growth parameters such as stem diameter and plant height were significantly influenced by various vermicompost treatments. The vermicompost of *P*. *cineraria* proved the most effective improving growth and yield attributes maize crop. The highest values of stem diameter, plant height, cob length, number of grains per cob, 1000-grain weight and grain yield were recorded with the application of *P*. *cineraria* vermicompost, whereas control treatment recorded the lowest values of these traits (Table 4).

**Table 4:** The impact of different vermicompost treatments on growth and yield attributes of maize crop.

Vermicompost source	Stem diameter (mm)	Plant height (cm)	Cob length (cm)	Number of grains/cob	1000-grain weight (g)	Grain yield t/ha
Absolute control	14.83 e	49.55 g	7.08	129.67 g	180.34 g	1.60 e
*Ziziphus mauritiana*	16.16 d	54.00 f	11.00 e	289.67 f	225.43 f	2.74 d
*Aerva javanica*	18.00 c	59.66 e	12.91 d	328.67 e	230.36 e	3.10 c
*Calligonum comosum*	20.08 b	65.00 d	15.16 c	340.00 d	241.30 d	3.09 c
*Sacchrum benghalens*	20.83 b	70.0 c	15.75 b	355.00 c	250.42 c	3.10 c
*Calligonum polygonoides*	21.03 b	72.57 b	16.08 b	360.00 b	255.48 b	3.15 b
*Prosopis cineraria*	22.66 a	75.33 a	17.66 a	374.67 a	260.41 a	3.20 a
LSD _(0.05)_	1.08	1.4	0.84	4.39	3.66	0.04

Means sharing the same letters within a column are statistically non-significant

Application vermicomposting enhances nutrient mobility; thus, plant uptakes more nutrient, which improves growth and yield attributes. Control plants resulted in the lowest stem diameter and plant height, which can be explained as a direct effect of nutrient availability. Results of this study are in line with several earlier work of [36–38].

The yield attributes, mainly yield and is the result of vegetative development of plant. All yield attributes were significantly influenced by vermicomposting of different desert species. These results have significantly attributed the importance of vermicomposting with different earthworm activities to increase the yield of several crops and improve defense mechanism against several pathogens and insects. Higher growth characters quantify higher yield attributes, particularly stem diameter and plant height, which ultimately lead to higher yield. Results of present study are supported by earlier studies [39, 40]. Improvement in cob length and number of grains/cob significantly improved yield in earlier studies [41–43].

The article "The influence of vermicomposting on photosynthetic activity and productivity of maize (Zea mays L.) crop under semi-arid climate" was retracted in 2022. Reasons: compromised peer review; a conflict of interest; concerns about the authorship.

### Nutrient uptake

Average yield potential is the result of co-ordinate interplay of different growth characters and nutrient uptake. Grain and stover yield is increased by increased nutrient uptake. The highest nutrient (N, P, K) uptake was observed with the application of *P*. *cineraria* vermicompost, whereas control treatment resulted in the lowest nutrient uptake (Table 5). Micronutrients and phenolic contents also increased with the application of vermicompost obtained from different plant species and *P*. *cineraria* (resulted in the highest values of micronutrients and phenolic contents (Table 5). Results of our study are in accordance with the findings of earlier studies [44–47]. The organic matter, i.e., FYM mainly supplies beneficial nutrients to crop and enhances its productivity significantly [48].

**Table 5:** The impact of different vermicompost treatments on the uptake of macro a d micronutrients.

Treatment combinations	N (%)	P (%)	K (%)	Micro-nutrients		
				Iron (ppm)	Zinc (ppm)	Phenolic contents
Absolute control	29.71 g	8.85 g	24.79 g	0.00 f	0.00 g	0.00 g
*Ziziphus mauritiana*	70.05 f	13.16 f	60.25 f	10.19 e	23.16 f	109.93 f
*Aerva javanica*	78.05 e	16.18 e	63.79 e	11.80 d	25.05 e	114.77 e
*Calligonum comosum*	80.71 d	17.70 d	65.06 d	15.04 c	30.05 d	120.05 d
*Sacchrum benghalens*	83.00 c	19.03 c	70.25 c	16.30 b	31.07 c	125.29 c
*Calligonum polygonoides*	86.96 b	20.31 b	75.05 b	16.65 b	35.05 b	140.08 b
*Prosopis cineraria*	91.01 a	22.07 a	80.41 a	19.07 a	40.05 a	150.00 a
LSD _(0.05)_	1.16	0.89	1.21	0.90	0.82	1.12

Means sharing the same letters within a column are statistically non-significant

### Physiological parameters of photosystem II

Physiological parameters of photosystem II, i.e., quantum photosynthetic yield (mol C/mole of photon) chlorophyll florescence (moles of photons m^-2^/S) and electron transport rate (μmolm^-2^S^-1^) were significantly altered by different vermicomposting treatments. The vermicompost of *P*. *cineraria* recorded the highest values of these traits, whereas the lowest values were recorded for control treatment (Table 6). Inappropriate function of photosynthetic apparatus may lead to less chlorophyll contents [49–51], and the application of vermicompost of *P*. *cineraria* and FYM improved photosynthetic parameters in the current study.

The article "The influence of vermicomposting on photosynthetic activity and productivity of maize (Zea mays L.) crop under semi-arid climate" was retracted in 2022. Reasons: compromised peer review; a conflict of interest; concerns about the authorship.

**Table 6:** The impact of different vermicompost treatments on quantum photosynthetic yield, chlorophyll florescence and electron transport rate.

Treatments	Quantum Photosynthetic Yield (mole C/mole of photon)	Chlorophyll Florescence (moles of photon m^-2^s^-1^)	Electron Transport Rate.(micro mole m^-2^s^-1^)
Absolute control	0.28 g	290.00 g	185.13 g
*Ziziphus mauritiana*	0.31 f	315.17 f	220.80 f
*Aerva javanica*	0.32 e	330.45 e	231.44 e
*Calligonum comosum*	0.34 d	332.97 d	234.56 d
*Sacchrum benghalens*	0.36 c	343.75 c	270.61 c
*Calligonum polygonoides*	0.40 b	344.34 b	272.42 b
*Prosopis cineraria*	0.42 a	355.18 a	310.18 a
LSD _(0.05)_	0.01	1.27	1.49

Means sharing the same letters within a column are statistically non-significant

Closure of stomata reduces internal concentration of CO_2_ and inhibits the functioning of Rubisco enzymes [52, 53], which mainly decrease the rate of photosynthesis. Numerous earthworm species utilize decaying organic materials and convert material to nutrient-rich elements, which further enhances vegetative and reproductive growth of plants [54]. However, very few studies have reported the role of vermicomposting on physiological parameters of photosystem II. Results of present study are also in line with the findings of [53, 55] that vermicomposting significantly increased chlorophyll contents, net photosynthetic rate and electron transport rate.

## Conclusion

It can be concluded that higher growth, nutrient uptake, quality and maximum yield potential can be achieved through combined application of vermicompost of *Prosopis cineraria* and FYM in maize. Results also proved that integrated nutrient management, i.e., application of vermicomposting strategies have multipurpose on the improvement of crop productivity in sustainable manners.

## Supporting information

S1 Dataset (XLSX)
